The article "Hsa-miR-139-5p inhibits proliferation and causes apoptosis associated with down-regulation of c-Met" was retracted in 2023. Reasons: duplicated images; signs of a paper mill; original data or images not available.

# Hsa-miR-139-5p inhibits proliferation and causes apoptosis associated with down-regulation of c-Met

**DOI:** 10.18632/oncotarget.5476

**Published:** 2015-10-14

**Authors:** Chengcao Sun, Ming Sang, Shujun Li, Xiaodong Sun, Cuili Yang, Yongyong Xi, Liang Wang, Feng Zhang, Yongyi Bi, Yunfeng Fu, Dejia Li

**Affiliations:** ^1^ Department of Occupational and Environmental Health, School of Public Health, Wuhan University, 430071 Wuhan, P.R.China; ^2^ Central Laboratory of the Fourth Affiliated Hospital in Xiangyang, College of Basic Medical Sciences, Hubei Key Laboratory of Wudang Local Chinese Medicine Research, Hubei University of Medicine, 442000 Shiyan, P. R. China; ^3^ Institute of Global Health, Wuhan University, 430071 Wuhan, P. R. China; ^4^ Wuhan Hospital for the Prevention and Treatment of Occupational Diseases, 430071 Wuhan, P. R. China; ^5^ The Third Xiang-ya Hospital of Central South University, 410013 Changsha, P. R. China

**Keywords:** Hsa-miRNA-139-5p (miR-139-5p), c-Met, non-small cell lung cancer (NSCLC), proliferation, apoptosis

## Abstract

Hsa-miRNA-139-5p (miR-139-5p) has recently been discovered having anticancer efficacy in different organs. However, the role of miR-139-5p on lung cancer is still ambiguous. In this study, we investigated the role of miR-139-5p on development of lung cancer. Results indicated miR-139-5p was significantly down-regulated in primary tumor tissues and very low levels were found in a non-small cell lung cancer (NSCLC) cell lines. Ectopic expression of miR-139-5p in NSCLC cell lines significantly suppressed cell growth through inhibition of cyclin D1 and up-regulation of p57(Kip2). In addition, miR-139-5p induced apoptosis, as indicated by up-regulation of key apoptosis gene cleaved caspase-3, and down-regulation of anti-apoptosis gene Bcl2. Moreover, miR-139-5p inhibited cellular metastasis through inhibition of matrix metalloproteinases (MMP)-7 and MMP-9. Further, oncogene c-Met was revealed to be a putative target of miR-139-5p, which was inversely correlated with miR-139-5p expression. Taken together, our results demonstrated that miR-139-5p plays a pivotal role in lung cancer through inhibiting cell proliferation, metastasis, and promoting apoptosis by targeting oncogenic c-Met.

## INTRODUCTION

MicroRNAs (miRNAs) are a class of small, highly conserved, and non-coding RNAs that regulate gene expression post-transcriptionally by binding to the 3′-untranslated region (3′-UTR) of target messenger RNAs (mRNAs) [1, 2]. More and more evidences suggest that miRNAs contribute to the transcription inhibition or translation of mRNA degradation. MiRNAs play vital roles in tumorigenesis by acting as tumor suppressors, such as let-7, miR-200 and miR-143 [3, 4] or oncogenes, such as miR-21, miR-155 and miR-95 [5–7]. Selective miRNA expression contributes to tumor proliferation, apoptosis, invasion, and metastasis, as well as anticancer drug resistance [8–10]. Though recent researches of miRNAs have brought mind-blowing insight into our knowledge of human cancers, there are still large amount of unknown details that need to be explored further.

The article "Hsa-miR-139-5p inhibits proliferation and causes apoptosis associated with down-regulation of c-Met" was retracted in 2023. Reasons: duplicated images; signs of a paper mill; original data or images not available.

Lung cancer has a higher death rate among all cancers, and is thus the leading cause of cancer-associated death. This trend is expected to continue until 2030. It is recognized as the leading cause of cancer-related deaths both in men and women in China, with an incidence of 3,372,175 new cases per year [11]. Approximately 80% of lung cancers are classified histopathologically as non-small cell lung carcinomas (NSCLC). At early stages of NSCLC, the only treatment is surgery, with a 5-year overall survival rate of 40% [12], whereas chemotherapy is mostly employed for small cell lung cancer (SCLC). These changes are attributed to silencing of tumor suppressor genes, dysregulation of proto-oncogenes, and an up-regulation of genes that promote cell growth and transformation and ultimately tumor development [13].

MiR-139-5p, a recognized tumor-suppressing miRNA, has been shown to be down-regulated in a variety of cancers, including gastric cancer, breast cancer and colorectal carcinoma [14]. Overexpression of miR-139-5p led to increase apoptosis, associated with caspase-3, caspase-7, and caspase-8 activities and expression of cytoplasm cytochrome C [15]. These data imply that miR-139-5p could play core roles in tumorigenesis. However, until now, there is no research investigating the role of miR-139-5p on development of lung cancer.

In this study, we investigated the role of miR-139-5p on the development of lung cancer. We show for the first time that miR-139-5p directly targets and regulates the full-length 3′-UTR of the human MET gene, which is up-regulated in many cancers, including lung cancer. c-Met is encoded by MET gene, and plays a key role in the control of invasive growth not only during tumorigenesis but also in embryonic development, organ development, and inflammatory response [16]. Here, we reported that miR-139-5p is indeed suppressed in primary lung cancers compared with the matching normal tissues, and found 3′-UTR of the human MET mRNA is really a target of miR-139-5p. Collectively, we discovered that miR-139-5p inhibits NSCLC cell growth, migration, invasion and colony formation, and promoted cell apoptosis by targeting 3′-UTR of c-Met.

## RESULTS

### MiR-139-5p is down-regulated in primary human lung cancer and NSCLC cell lines

To determine whether miR-139-5p is down-regulated in lung cancer, we measured the mature miR-139-5p level in human primary lung tumors (NSCLC) and pair-matched adjacent lung normal tissues by qRT-PCR. We used U6 that is not deregulated in lung cancer for normalization. The results showed that miR-139-5p expression in the tumors was significantly (*P* < 0.05) reduced in 13 lung cancers relative to their matched controls among 13 samples analyzed (Figure 1A). Next, we examined miR-139-5p expression in NSCLC cell lines, and results demonstrated a lower expression of miR-139-5p in A549 and SK-MES-1 cell lines, compared with that of in normal lung cells HELF (Figure 1A). Additionally, Kaplan–Meier survival analysis revealed that patients with low expression levels of miR-139-5p had shorter overall survival, when compared with patients with high expression levels of miR-139-5p (Figure 1B). These results show that down-regulated miR-139-5p is associated with poor prognosis. Thus, it was concluded that the decreased expression of miR-139-5p might play an important role in lung cancer progression and development.

The article "Hsa-miR-139-5p inhibits proliferation and causes apoptosis associated with down-regulation of c-Met" was retracted in 2023. Reasons: duplicated images; signs of a paper mill; original data or images not available.

**Figure 1:** Expression miR-139-5p is significantly down-regulated in primary human lung cancer and NSCLC cell lines **A.** Left. miR-139-5p is significantly decreased in primary human lung cancer tissues in comparison to matched-normal lung cancer tissues. *n* = 13 for each group. Right. The expression level of miR-139-5p in two NSCLC cell lines and normal HELF cells. Assays were performed in triplicate. **B.** Kaplan-Meier survival analysis revealed that down-regulated miR-139-5p is associated with poor prognosis in patients with non-small cell lung cancer. Means ± SEM are shown. Statistical analysis was conducted using student *t*-test.

### Inhibition of miR-139-5p does not reverse the anticancer efficacy of silence of MET expression *in vitro*

We next examined the potential tumorigenicity of MET in lung cancer. Silence of MET expression by siRNA significantly inhibited the expression of c-Met (Figure 2A). Moreover, loss of MET expression also contributed to inhibition of lung cancer cell (both A549 and SK-MES-1 cells) growth (Figure 2B and 2C) and migration (Figure 2D and 2E). In addition, inhibition of MET expression promoted apoptosis in lung cancer cell (both A549 and SK-MES-1 cells) (Figure 2F). These results further verified the powerful tumorigenicity of MET in lung cancer. Thus, we adopted MET for as targeted oncogenes. However, inhibition of miR-139-5p does not reverse the anticancer efficacy of silence of MET expression in lung cancer cell (both A549 and SK-MES-1 cells). These results indicate that the anticancer efficacy of miR-139-5p is partly attributed to its inhibitory role on c-met.

The article "Hsa-miR-139-5p inhibits proliferation and causes apoptosis associated with down-regulation of c-Met" was retracted in 2023. Reasons: duplicated images; signs of a paper mill; original data or images not available.

**Figure 2:** Silence of MET expression inhibits lung cancer cell growth, migration, invasion and apoptosis **A.** Western blot of c-Met protein in siRNA MET treated and blank A549 and SK-MES-1 cells. **B.** CCK8 assays of A549 and SK-MES-1 cells after transfected (un-transfected) with siRNA MET. **C.** Shown are representative photomicrographs of colony formation assay after transfected with (without) siRNA MET for ten days. **D.** Shown are representative photomicrographs of transwell migration assay after transfected with (without) siRNA MET. **E.** Shown are representative photomicrographs of transwell invasion assay after transfected with (without) siRNA MET. **F.** Quantitative representation of caspase-3 activity in A549 and SK-MES-1 cells transfected with (without) siRNA MET for forty-eight hours. Assays were performed in triplicate. Means ± SEM are shown. Statistical analysis was conducted using One-way ANOVA.

### MiR-139-5p inhibits lung cancer cell proliferation and colony formation

To further investigate the anticancer role of miR-139-5p in lung cancer, we transfected A549 and SK-MES-1 cells with miR-139-5p mimic or miR mimic NC, and miR-139-5p inhibitor or miR-139-5p inhibitor NC, separately. As expected, miR-139-5p mimic significantly increased the expression of miR-139-5p, while miR-139-5p inhibitor inhibited it (Supplementary Figure S1A). Then, we examined the role of miR-139-5p on A549 and SK-MES-1 cells proliferation. Our results of BrdU staining revealed that miR-139-5p inhibited A549 and SK-MES-1 cells growth by approximately 78% and 82% (Supplementary Figure S1B–S1E), compared with blank A549 and SK-MES-1 cells, respectively. However, miR-139-5p inhibitor treatment increased A549 and SK-MES-1 cells growth by approximately 1.5 and 2 folds, compared with blank A549 and SK-MES-1 cells (Supplementary Figure S1B–S1E). To verify this result, we also did the CCK8 assay, and results demonstrated that miR-139-5p significantly promoted A549 and SK-MES-1 cells proliferation, while loss of miR-139-5p attenuated it (Figure 3A). In addition, we used colony formation assay to investigate the role of miR-139-5p on clonogenic survival. MiR-139-5p mimic treatment caused a decrease in the clonogenic survival of A549 cells compared with blank A549 cells (Figure 3B and 3D), while miR-139-5p inhibitor-treated A549 showed a significant increase in the clonogenic survival of A549 cells compared with blank A549 cells (Figure 3B and 3C).

**Figure 3:** Ectopic expression of miR-139-5p inhibits NSCLC cell growth A549 and SK-MES-1 cells were transfected with miR-139-5p mimic and mimic NC, miR-139-5p inhibitor and inhibitor NC, for forty-eight hours, respectively. **A.** CCK8 assays of A549 and SK-MES-1 cells after transfection. **B.** Shown are representative photomicrographs of colony formation assay in A549 and SK-MES-1 cells after transfection. **C.** Statistical analysis of colony formation assay. **D.** Western blot of cyclin D1 protein in A549 and SK-MES-1 cells after transfection. **E.** Upper, statistical analysis of Western blot; Lower, qRT-PCR of cyclin D1 mRNA in A549 cells after transfection. **F.** qRT-PCR of p57 mRNA in A549 and SK-MES-1 cells after transfection. Assays were performed in triplicate. Means ± SEM are shown. Statistical analysis was conducted using One-way ANOVA.

The article "Hsa-miR-139-5p inhibits proliferation and causes apoptosis associated with down-regulation of c-Met" was retracted in 2023. Reasons: duplicated images; signs of a paper mill; original data or images not available.

We next examined the influence of miR-139-5p on the expression of cyclin D1, which is overexpressed in a significant proportion of human cancers including breast, prostate and lung cancer [19], and promotes cell growth in most of tumors. Our results discovered that the protein and mRNA of cyclin D1 was higher expressed in lung cancer tissues than the adjacent normal lung tissues (Supplementary Figure S1F). In addition, we also found that miR-139-5p significantly decreased the protein and mRNA expression of cyclin D1, while loss of miR-139-5p remarkably increased the level of cyclin D1 in A549 cells (Figure 3D and 3E). p57 is a cyclin-dependent kinase inhibitor, and it is considered to be a candidate of tumor suppressor gene that has been implicated in cancers [20]. Our study revealed that the over-expression of miR-139-5p is a mechanism for the up-regulation of p57 level in NSCLC cell lines (A549 and SK-MES-1) (Figure 3F).

Collectively, these results clearly revealed that miR-139-5p markedly inhibited cell growth in lung cancer cells.

### MiR-139-5p inhibits lung cancer cell migration and invasion

Then, we examined the role of miR-139-5p on A549 cells migration and invasion. Invasion and migration through the basement membrane are characteristics of metastatic cancer cells. We used two different approaches to assess the role of miR-139-5p on the ability of A549 and SK-MES-1 cells migration. In the first technique, we used a “scratch wound healing” assay. Motility of cells at different time points after generation of the wound was monitored under a microscope. Closure of the wound was nearly complete within forty-eight hours in control A549 cells. In contrast, miR-139-5p-expressing cells migrated toward the wound at a much slower rate (Figure 4A and 4B). Loss of miR-139-5p significantly promoted cells migrated toward the wound at a faster rate (Figure 4C and 4D). In the second approach, cells were seeded in serum-free medium on the top chamber of a two-chamber trans-well cell culture plate, and the cells migrated to the lower chamber containing complete medium after twenty-four hours were photographed and counted. As expected, migration of miR-139-5p-expressing clones was inhibited by 65% in A549 cells and by 53% in SK-MES-1 cells, compared with the blank A549 and SK-MES-1 cells, respectively (Figure 4E and 4F, 4I and 4J). Colorimetric estimation of migrated cells showed 70% and 35% decrease in miR-139-5p mimic treated A549 and SK-MES-1 cells, compared with the blank A549 and SK-MES-1 cells, respectively (Figure 4F and 4J). However, when treated with miR-139-5p inhibitor, migration in miR-139-5p-expression defect A549 cells and SK-MES-1 cells were significantly increased, relative to blank A549 and SK-MES-1 cells, respectively (Figure 4E and 4F, 4I and 4J).

The article "Hsa-miR-139-5p inhibits proliferation and causes apoptosis associated with down-regulation of c-Met" was retracted in 2023. Reasons: duplicated images; signs of a paper mill; original data or images not available.

**Figure 4:** Ectopic expression of miR-139-5p in A549 and SK-MES-1 cells reduces cell migration and invasion motility A549 and SK-MES-1 cells were transfected with miR-139-5p mimic and mimic NC, miR-139-5p inhibitor and inhibitor NC, for forty-eight hours, respectively. **A.** Shown are representative photomicrographs of “wound healing assay” in A549 cells after transfected with miR-139-5p mimic and mimic NC for twenty-four hours and forty-eight hours. Bar = 100 μm. **B.** Statistical analysis of “wound healing assay”. **C.** Shown are representative photomicrographs of “wound healing assay” in A549 cells after transfected with miR-139-5p inhibitor and inhibitor NC for twenty-four hours and forty-eight hours. Bar = 100 μm. **D.** Statistical analysis of “wound healing assay”. **E.** A549 cells were loaded onto the top well of a transwell inserts for cell migration assay. After twenty-four hours, cells that migrated to the bottom chamber containing serum-supplemented medium were stained with 0.1% crystal violet, visualized under a phase-contrast microscope, and photographed. Bar = 50 μm. **F.** Upper, total number of cells in five fields was counted manually; Lower, 0.1% crystal violet-stained cells were solubilized in 33% acetic acid, and absorbance was measured at 570 nm. **G.** A549 cells were loaded onto the top well of a transwell inserts for cell invasion assay. After twenty-four hours, cells that migrated to the bottom chamber containing serum-supplemented medium were stained with 0.1% crystal violet, visualized under a phase-contrast microscope, and photographed. Bar = 50 μm. **H.** Upper, total number of cells in five fields was counted manually; Lower, 0.1% crystal violet-stained cells were solubilized in 33% acetic acid, and absorbance was measured at 570 nm. **I.** SK-MES-1 cells were loaded onto the top well of a transwell inserts for cell migration assay. After twenty-four hours, cells that migrated to the bottom chamber containing serum-supplemented medium were stained with 0.1% crystal violet, visualized under a phase-contrast microscope, and photographed. Bar = 50 μm. **J.** Upper, total number of cells in five fields was counted manually; Lower, 0.1% crystal violet-stained cells were solubilized in 33% acetic acid, and absorbance was measured at 570 nm. **K.** SK-MES-1 cells were loaded onto the top well of a transwell inserts for cell invasion assay. After twenty-four hours, cells that migrated to the bottom chamber containing serum-supplemented medium were stained with 0.1% crystal violet, visualized under a phase-contrast microscope, and photographed. Bar = 50 μm. **L.** Upper, total number of cells in five fields was counted manually; Lower, 0.1% crystal violet-stained cells were solubilized in 33% acetic acid, and absorbance was measured at 570 nm. **M.** Expression of MMP-9 mRNA in A549 and SK-MES-1 cells after transfection. **N.** Expression of MMP-7 mRNA in A549 and SK-MES-1 cells after transfection. Assays were performed in triplicate. Means ± SEM are shown. Statistical analysis was conducted using One-way ANOVA.

The article "Hsa-miR-139-5p inhibits proliferation and causes apoptosis associated with down-regulation of c-Met" was retracted in 2023. Reasons: duplicated images; signs of a paper mill; original data or images not available.

To investigate the role of miR-139-5p on A549 cells invasion, we used a transwell invasion assay. As expected, invasion of miR-139-5p-expressing clones was inhibited by 75% in A549 cells and by 60% in SK-MES-1 cells, relative to the blank A549 and SK-MES-1 cells, respectively (Figure 4G and 4H, 4K and 4L). Colorimetric estimation of migrated cells showed 50% and 45% decrease in miR-139-5p mimic treated A549 and SK-MES-1 cells, compared with the blank A549 and SK-MES-1 cells, respectively (Figure 4H and 4L). However, when treated with miR-139-5p inhibitor, invasion in miR-139-5p-expression defect A549 cells were significantly increased, relative to blank A549 and SK-MES-1 cells (Figure 4G and 4H, 4K and 4L).

We also investigated the role of miR-139-5p on expression of MMP-9 and MMP-7, which all play a key role on tumor metastasis, and results indicated miR-139-5p inhibited the mRNA expression of MMP-9 and MMP-7 both in A549 and SK-MES-1 cells (Figure 4M and 4N). As expected, loss of miR-139-5p significantly increased the mRNA expression of MMP-9 and MMP-7 in both A549 and SK-MES-1 cells (Figure 4M and 4N).

Taken together, these results clearly demonstrated that miR-139-5p expression markedly reduces the migration and invasion motility of lung cancer cells.

### MiR-139-5p promotes lung cancer cell apoptosis

Next, we examined the role of miR-139-5p on A549 and SK-MES-1 cells apoptosis. Hoechst 33342 staining revealed that miR-139-5p significantly increased the number of apoptosis cells in A549 and SK-MES-1 cells, while inhibition of miR-139-5p attenuated DNA damaging and nuclear fragmentation both in A549 and SK-MES-1 cells (Figure 5A–5D). Moreover, we also use dual-staining of annexin/PI to further evaluate the positive role of miR-139-5p in apoptosis of A549 cells. We found that miR-139-5p significantly promoted apoptosis in A549 cells, while inhibition of miR-139-5p reversed the high level of apoptosis in comparison with miR-139-5p treated A549 cells (Figure 5E). Further, our results of flow cytometric analysis demonstrated that forced expression of miR-139-5p resulted in a ~4-fold increase in apoptotic cell death of A549 cell (Figure 5F and 5G), while the percentage of apoptotic cells induced by miR-139-5p was decreased to the basal level when the cells were treated with the specific miR-139-5p inhibitor (Figure 5F and 5G). Induction of apoptosis was further confirmed by the expression of apoptosis-related protein using western blot. As shown in Figure 5J and 5K, the protein levels of the active forms of caspase-3 was enhanced in miR139-5p treated A549 cells, compared with blank A549 cells, while inhibition of miR-139-5p significantly decreased the expression of casepase-3 (Figure 5J and 5K). In addition, we tested the caspase-3 activity after treated A549 and SK-MES-1 cells with miR-139-5p mimic or miR-139-5p mimic NC, miR-139-5p inhibitor or miR-139-5p inhibitor NC, and results showed that miR-139-5p significantly increased the caspase-3 activity in A549 and SK-MES-1 cell lysate, by approximately 8 folds and 4.5 folds increase than that of bank A549 and SK-MES-1 cells, respectively (Figure 5L). However, loss of miR-139-5p by transfecting with miR-139-5p inhibitor remarkably reduced the caspase-3 activity in A549 and SK-MES-1 cell lysate, by approximately 64% and 50% than that of bank A549 and SK-MES-1 cells (Figure 5L). We also investigated the role of miR-139-5p on expression of Bcl2, a vital anti-apoptosis protein *in vivo* and vitro. Our results revealed that miR-139-5p significantly inhibited the protein and mRNA expression in A549 cells, while inhibition of miR-139-5p remarkably promoted the protein and mRNA expression in A549 cells (Figure 5H and 5I). These results demonstrated that miR-139-5p indeed promoted apoptosis in A549 cells.

The article "Hsa-miR-139-5p inhibits proliferation and causes apoptosis associated with down-regulation of c-Met" was retracted in 2023. Reasons: duplicated images; signs of a paper mill; original data or images not available.

**Figure 5:** Ectopic expression of miR-139-5p promotes apoptosis in A549 and SK-MES-1 cells A549 and SK-MES-1 cells were transfected with miR-139-5p mimic and mimic NC, miR-139-5p inhibitor and inhibitor NC, for forty-eight hours, respectively. **A.** Shown are representative photomicrographs of A549 cells stained with Hoechst. Cells grown in coverslips were stained with Hoechst 33342 and photographed under a fluorescence microscope. Cells undergoing DNA fragmentation were counted manually. Bar = 50 μm. **B.** Quantitative representation of the number of apoptotic after transfecting cells with related miRNAs for forty-eight hours. The total number of cells (~200) with or without fragmented nuclei was counted, and the percentage of apoptotic cells was calculated. **C.** Shown are representative photomicrographs of SK-MES-1 cells stained with Hoechst. Cells grown in coverslips were stained with Hoechst 33342 and photographed under a fluorescence microscope. Cells undergoing DNA fragmentation were counted manually. Bar = 50 μm. **D.** Quantitative representation of the number of apoptotic after transfecting cells with related miRNAs for forty-eight hours. The total number of cells (~200) with or without fragmented nuclei was counted, and the percentage of apoptotic cells was calculated. **E.** Shown are representative photomicrographs of cells dual-stained with annexin-FITC/PI. Bar = 5 μm. **F.** Shown are representative photomicrographs of flow cytometric analysis. **G.** Statistical analysis of flow cytometric analysis. **H.** Expression of Bcl2 protein in transfected A549 cells. Western blot of Bcl2 protein in A549 cells after transfection. **I.** Upper, statistical analysis of Western blot; Lower, qRT-PCR of Bcl2 mRNA in A549 cells after transfection. **J.** Western blot of cleaved-caspase-3 and caspase-3 (total) protein in A549 cells after transfection. **K.** Statistical analysis of Western blot. **L.** Quantitative representation of caspase-3 activity in A549 Upper, and SK-MES-1 Lower, cells transfected with related miRNAs for forty-eight hours. Assays were performed in triplicate. Means ± SEM are shown. Statistical analysis was conducted using One-way ANOVA.

### MiR-139-5p targets human MET

We then explored the underlying molecular mechanism of the antitumorigenic property of miR-139-5p in lung cancer cells. We first examined c-Met expression in human primary lung tumors (NSCLC) and pair-matched lung tissues, and our western blot results demonstrated that the expression of c-Met protein was increased in lung cancer tissues compared with normal lung tissues (Figure 6A). These results were confirmed by qRT-PCR of c-Met mRNA expression (Figure 6A). Since miRNAs primarily mediate their biological functions in animal cells by impeding the expression of target genes, we searched different data bases (TargetScan, http://microRNA.org and PicTar) for its potential targets that exhibited oncogenic properties. MET (hepatocyte growth factor receptor), which harbors one conserved miR-139-5p cognate site (Figure 6C), is a predicted target of miR-139-5p. To determine whether MET expression are indeed regulated by miR-139-5p, the MET was cloned into a luciferase reporter plasmid (Figure 6B), and the ability of miR-139-5p to inhibit expression of the adjacent hRluc coding region was quantified. For this purpose, the luciferase reporter plasmid pmiR-RB-REPORT™ -MET-3′-UTR or a mutant reporter plasmids carrying point mutations in the putative miR-139-5p binding sites was co-transfected with miR-139-5p mimics or miR mimic NC, separately. The results show that miR-139-5p suppresses luciferase activity by approximately 55% when the reporter plasmid carried the wild type MET 3′-UTR (Figure 6D, *p* < 0.05), but no significant suppression was observed when the reporter plasmid carried a mutant MET 3′-UTR (i.e., pmiR-RB-REPORT™-mut-MET-3′ -UTR). Moreover, we evaluated the correlation between MET mRNA and miR-139-5p expression in 13 lung cancer tissues. Expression of MET mRNA and miR-139-5p exhibited a significant inverse correlation as calculated by Pearson correlation (*r* = − 0.0748, *P* = 0.0038) (Figure 6E), which further supported that miR-139-5p targeted to MET. We next examined the role of miR-139-5p on the expression of c-Met. Our results of western blot demonstrated that miR-139-5p inhibited expression of c-Met protein by 58%, when compared with blank A549 cells (Figure 6F and 6G). Interestingly, we also found that miR-139-5p also decreased the mRNA of c-Met (Figure 6F and 6G). We assumed that miR-139-5p might play a role on regulation of the upstream of c-Met, thus we detected the protein expression of HGF (the ligand of c-Met and c-Met was activated by HGF), and results demonstrated that miR-139-5p suppressed the protein expression of HGF (Supplementary Figure S2A). The decrease of expression of HGF by treating with miR-139-5p may contribute to the lower mRNA levels of c-Met. However, as expected, inhibition of miR-139-5p increased protein and mRNA expression in A549 cells, relative to blank A549 cells (Figure 6F and 6G). In addition, our immunofluorescence of c-Met also demonstrated that miR-139-5p reduced the expression of c-Met in A549 cells, and inhibition of miR-139-5p significantly promoted c-Met expression (Figure 6H and Supplementary Figure S2B). These results suggest that miR-139-5p binds directly to the predicted binding site(s) in the MET 3′-UTR and negatively regulates MET expression.

The article "Hsa-miR-139-5p inhibits proliferation and causes apoptosis associated with down-regulation of c-Met" was retracted in 2023. Reasons: duplicated images; signs of a paper mill; original data or images not available.

**Figure 6:** Oncogene MET is a target of miR-139-5p at specific 3′-UTR site Assays were performed in triplicate. Means ± SEM are shown. Statistical analysis was conducted using One-way ANOVA. **A.** Western blot of c-Met protein and qRT-PCR of c-Met mRNA expression in lung cancer tissues and normal lung cancers. **B.** pmiR-RB-REPORT™ dual-luciferase reporter vector. **C.** The 3′-UTR of MET harbor one miR-139-5p cognate site. **D.** Relative luciferase activity of reporter plasmids carrying wild-type or mutant MET 3′-UTR in A549 and SK-MES-1 cells co-transfected with negative control (NC) or miR-139-5p mimic. **E.** Scatter plots showing the inverse association between miR-139-5p level and MET mRNA expression. **F.** Western blot of c-Met(total) and phospho-c-Met protein in A549 cells after transfection. **G.** Upper, statistical analysis of Western blot; Lower, qRT-PCR of c-Met mRNA in A549 cells after transfection. **H.** c-Met immune-staining in A549 cells after transfection. Assays were performed in triplicate. Means ± SEM are shown. Statistical analysis was conducted using One-way ANOVA.

### MiR-139-5p suppresses tumor growth *in vivo*

To confirm the tumor suppressor role of miR-195-5p *in vivo*, we established a BALB/c nude mouse xenograft lung cancer model using A549 cells. After 8 days, miR-195-5p agomir or miR agomir NC was directly injected into the implanted tumor every 4 days for seven times. The tumor volume was measured every 4 days until day 36. The tumor volume and weight of mice treated with miR-195-5p agomir were significantly reduced relative to miR agomir NC (Figure 7A and 7B). This result indicates that miR-195-5p significantly inhibits the tumorigenicity of A549 cells in the nude mouse xenograft model. Western blot and qRT-PCR demonstrated the decreased expression of c-Met in tumors developed from miR-195-5p-agomir-treated nude mice relative to control tumors (Figure 7C and 7D).

**Figure 7:** Ectopic expression of miR-139-5p suppresses tumor growth *in vivo* **A–B.** Tumor volume and weight in nude mice. Each group contained six mice (*n* = 6); the data are presented as the mean ± SEM; *p < 0.001, compared with the NC group. **C.** The expression of c-Met protein in nude mice. **D.** The expression of c-Met mRNA in nude mice. Assays were performed in triplicate. Means ± SEM are shown. Statistical analysis was conducted using student *t*-test.

## DISCUSSION

Although dysregulation of miRNAs was reported in various types of human cancers [21], aberrant expression and potential role of miRNAs in lung cancers were under studied. Down-regulation of miR-139-5p has been reported by miRNA profile studies on gastric cancer [22], colorectal cancer [23], endometrial serous adenocarcinoma [24] and HCC [25]. Our data also indicated that miR-139-5p showed a reduced expression in lung cancer, suggesting the dysregulation of miR-139-5p is an early event of lung tumorigenesis.

The article "Hsa-miR-139-5p inhibits proliferation and causes apoptosis associated with down-regulation of c-Met" was retracted in 2023. Reasons: duplicated images; signs of a paper mill; original data or images not available.

We therefore characterized the putative tumor suppressive function of miR-139-5p in human NSCLC cell lines. We found that the restoration of miR-139-5p in NSCLC cell lines A549 and SK-MES-1 significantly inhibited cell proliferation as evidenced by cell viability and colony formation assays. Previous study suggested that miR-139-5p did not affect the proliferation phenotype and DNA profile of breast cancer cell MDA-MB-231 based on Doxycycline-induced plasmid expression [26]. However, miR-139-5p shows an anti-proliferative effect in lung cancer. This discrepancy may be attributed to a tissue specific function of miR-139-5p signaling in NSCLC compared with other solid tumors.

Then we examined the mechanism of miR-139-5p on lung cancer cell growth, and found that over-expression of miR-139-5p significantly inhibited A549 and SK-MES-1 cell proliferation, while loss of miR-139-5p promoted cell growth in A549 and SK-MES-1 cells. The growth-inhibition role of miR-139-5p may attribute to that miR-139-5p targets 3′-UTR of MET mRNA, and inhibits the expression of MET in lung cancer cells. In addition, miR-139-5p also inhibited cyclin D1 and promoted p57 expression levels in lung cancer cells, which further contributed to the growth-delay efficacy of miR-139-5p.

In the present work, we showed that, in addition to inhibition of cell proliferation, the growth inhibitory effect of miR-139-5p was also related to induction of apoptosis. We observed that induction of miR-139-5p mediated apoptosis occurs by the modulation of extrinsic apoptosis pathway. Apoptosis induced by extrinsic pathways has been considered to be an important antitumor mechanism [27–29]. After transfection with miR-139-5p, the expression of vital anti-apoptosis protein Bcl2 was down-regulated, and the activity of the downstream active apoptosis executor caspase-3 was up-regulated, leading to initiate a caspase cascade, and causing loss of DNA repair, cellular disassembly and finally apoptosis.

*In vitro* assays showed that re-expression of miR-139-5p inhibited the cell migration and invasive capabilities. The reduced spreading effect and cell motility caused by miR-139-5p in lung cancer cells was revealed to be associated with the inhibition of the protein expression of cell migration and invasion molecules MMP-7 and MMP-9. MMP-7 and MMP-9 are members of the matrix metalloproteinases (MMPs) family, which are extracellular proteinases that regulate basic cellular processes including survival, migration and morpho-genesis and degradation extracellular matrix during the cancer metastatic process [30, 31]. MMP-7 is an established instigator of aggressive behavior in a number of cancer types including NSCLC. MMP-9 has been identified as a critical component for priming of the pre-metastatic niche. Thus, down-regulation of MMP-7 and MMP-9 expression by miR-139-5p contributed to dampened cell spreading and invasion ability.

The article "Hsa-miR-139-5p inhibits proliferation and causes apoptosis associated with down-regulation of c-Met" was retracted in 2023. Reasons: duplicated images; signs of a paper mill; original data or images not available.

Epigenetic silencing of miRNAs with tumor suppressor features is a common hallmark of human tumors. Having shown the crucial role of miR-139-5p in suppressing NSCLC development, we sought for the possible gene effectors participating in its function. Of note, a single miRNA can regulate a multitude of target genes concomitantly; for instance, it has been reported that miR-139-5p suppresses progression of liver cancer by down-regulating Rho-kinase 2 [32]; and miR-139-5p could repress the activity of RAP1B [33] and IGF-IR [34] in colon cancer. Among the miRNAs predicted to target genes, we found that c-Met acts as a critical effector of miR-139-5p. We showed that miR-139-5p was able to significantly repress the luciferase activity of Luc-MET-3′UTR by targeting the 3′UTR of c-Met mRNA. Therefore we focused on c-Met for further analysis.

MET is a receptor for hepatocyte growth factor and a tyrosine kinase (receptor-type tyrosine kinase), and supports the initial steps of invasion and metastasis of most human cancers, including lung cancer [35]. The down-regulation of MET could be a possible mechanism by which miR-139-5p regulates growth and metastatic potential of these cells. c-Met is encoded by MET gene, and plays a key role in the control of invasive growth not only during tumorigenesis but also in embryonic development, organ development, and inflammatory response [16]. Aberrantly activated MET signaling has been observed during the carcinogenesis of several human cancers, including lung cancer [36–41]. We observed that the expression level of c-met was inversely correlated with miR-139-5p expression in NSCLC patients, suggesting miR-139-5p potentially inhibits c-met gene and mRNA expression (Figure 5A). Moreover, we revealed that expression of MET mRNA and miR-139-5p exhibited a significant inverse correlation as calculated by Pearson correlation (*r* = −0.0748, *P* = 0.0038) (Figure 5E). We also demonstrated that c-Met levels directly down-regulated by introduction of miR-139-5p in NSCLC cells (Figure 5F and 5G). This result further supported that miR-139-5p targeted to MET. In agreement with our results, it has been shown that suppression of MET inhibits tumor growth in human hepatocellular carcinomas [41] and in breast cancer [40] by regulating cell proliferation and cycle.

Recent studies have reported that miR-139-5p was a potential prognostic marker for renal cell carcinoma and endometrial serous adenocarcinoma [42, 43]. The clinical value of miR-139-5p in NSCLC is still controversial. In our study, we have shown that miR-139-5p is dramatically down-regulated in human lung cancer tissues compared with normal lung tissues. Moreover, up-regulation of miR-139-5p suppresses lung cancer cell growth and metastasis, and promotes lung cancer cell apoptosis, through targeting c-Met. Our experimental data may provide a strategy for targeting the miR-139-5p/c-Met interaction in a novel therapeutic application to treat lung cancer patients.

The article "Hsa-miR-139-5p inhibits proliferation and causes apoptosis associated with down-regulation of c-Met" was retracted in 2023. Reasons: duplicated images; signs of a paper mill; original data or images not available.

## MATERIALS AND METHODS

### Tissue collection

Lung cancer tissues and adjacent normal lung tissues were obtained from patients who had undergone surgery at the People's Hospital of Wuhan University, between 2013 and 2015 and who were diagnosed with lung cancer based on histopathological evaluation. No local or systemic treatment had been conducted in these patients before the operation. All the tissue samples were collected, immediately snap frozen in liquid nitrogen, and stored at −80°C until RNA extraction. The study was approved by the Research Ethics Committee of Wuhan University (Wuhan, Hubei, PR China). Informed consent was obtained from all patients.

### Cell culture and transfection

The human NSCLC cell lines, namely, A549 and SK-MES-1, were grown in RPMI 1640 or DMED medium (Gibco, USA) containing 10% heat-inactivated (56°C, 30 min) fetal calf serum, 2 mmol/L glutamine, penicillin (100 U/mL) and streptomycin (100 U/mL), which was maintained in an incubator at 37°C with 5% CO2 in a humidified atmosphere. Hsa-miRNA-139-5p mimic and mimic negative control, Hsa-miRNA-139-5p inhibitor and inhibitor negative control were purchased from RiboBio Co., Ltd. (Guangzhou, China). For convenience, Hsa-miRNA-139-5p mimic and mimic negative control, Hsa-miRNA-139-5p inhibitor and inhibitor negative control were simply referred to as miR-139-5p mimic and miR mimic NC, miR-139-5p inhibitor and miR inhibitor NC, respectively. Complete medium without antibiotics was used to culture the cells at least twenty-four hours prior to transfection. The cells were washed with 1× PBS (pH7.4) and then transiently transfected with 50 nM miR-139-5p mimic or miR mimic NC, 100 nM miR-139-5p inhibitor or miR inhibitor NC, using Lipofectamine™ 2000 (Invitrogen, Carlsbad, CA, USA) according to the manufacturer's instructions.

### Western blot analysis

Forty-eight hours after transfection, total protein was extracted from the A549 and SK-MES-1 cells using RIPA cell lysis reagent containing proteinase and phosphatase inhibitors (Solarbio) at 4°C for 30 min. Cell lysates were centrifuged at 12,000 × g for 20 min at 4°C, and the protein concentrations of the supernatant were determined using the BCA protein assay reagent kit (Beyotime) [17, 18]. The supernatants containing total protein were then mixed with a corresponding volume of 5 × SDS loading buffer and heated at 100°C for 10 min. Then, the supernatant lysates were run on 10% SDS-polyacrylamide gels (50 μg/lane), and proteins were transferred to poly (vinylidene fluoride) (PVDF) membranes (Hertfordshire, UK) by semidry electroblotting (1.5 mA/cm2). PVDF membranes were then incubated in blocking buffer [Tris-buffered saline (TBS) supplemented with 0.05% (vol/vol) Tween 20; TBST] containing 5% (wt/vol) skimmed milk powder for 120 min at room temperature followed by three 10 min washes in TBST. The PVDF membranes were then incubated with anti-c-Met (1:1000 dilutions, Affinity), anti-phospho-c-Met (1:1000 dilutions, Affinity), anti-Bcl2 (1:1,000 dilutions, Affinity), anti-caspase 3 (1:1,000 dilutions, Affinity), anti-cleaved caspase 3 (1:1,000 dilutions, Affinity), anti-cyclin D1 (1:1,000 dilutions, Affinity) and anti-GADPH (1:5,000 dilutions, Affinity) as internal normalizers in TBST containing 5% (wt/vol) skimmed milk powder (antibody buffer) overnight at 4°C on a three-dimensional rocking table. Then the membranes were washed three times for 10 min in TBST and then incubated with goat anti-rabbit IgG conjugated to horseradish peroxidase (1:12,000 dilutions) in antibody buffer for 120 min. Finally, membranes were washed three times for 10 min in TBST and exposed to ECL Advance reagent (GE Healthcare Biosciences, Buckinghamshire, UK) for 2 min as described in the manufacturer's protocol. Then membranes were exposed to Hyperfilm-ECL (GE Healthcare Bio-Sciences) for 2–5 min and visualized using a Fluor S Multimager and Quantity One 4.1 (Bio-Rad Laboratories, Hercules, CA). The molecular weights of the bands were calculated by a comparison with prestained molecular weight markers (molecular weight range: 6,500–250,000) that were run in parallel with the samples. Semiquantitative analysis of specific immunolabeled bands was performed using a Fluor S image analyzer and Quantity One 4.1.

The article "Hsa-miR-139-5p inhibits proliferation and causes apoptosis associated with down-regulation of c-Met" was retracted in 2023. Reasons: duplicated images; signs of a paper mill; original data or images not available.

### RNA isolation and quantitative reverse transcription poly-merase chain reaction (qRT-PCR)

Total RNA from the cultured cells was extracted using Trizol reagent (Invitrogen) according to the manufacturer's instructions. MiRNA levels were measured by qRT-PCR. For the qRT-PCR detection of mature miR-139-5p expression, we purchased the Bulge-Loop™ miRNA qRT-PCR Primer Set and the miRNA qRT-PCR Control Primer Set (both from RiboBio). RNA (2 μg) was converted into cDNA using the PrimeScript™ RT reagent kit with gDNA Eraser (Takara, Dalian, China) according to the manufacturer's instructions. qRT-PCR was performed using SYBR^®^ Premix Ex Taq™ II (Takara) in the ABI PRISM^®^ 7300 real-time PCR system (Applied Biosystems, Foster City, CA, USA). GADPH and U6 were used as endogenous controls. In addition, melting curves were used to evaluate non-specific amplification. The relative expression level was calculated using the 2™ΔΔCt method. The primer sequences used in this study are presented in Table 1 and 2. The formula and its derivations were obtained from the ABI Prism 7300 sequence detection system user guide. Statistical analysis was performed on the fold change.

**Table 1:** Primer sequences for quantitative reverse transcription (RT)-PCR (miRNA)

miRNA	Sequence (5′ → 3′)
**miR-139-5p**	Reverse-transcribed primer: 5′-GTCAGAAGGAATGATGCACAGCCACTGGAG-3′
	Forward:5′-TCTACAGTGCACGTGTCTCCAG-3′ Reverse:5′-ACCTGCGTAGGTAGTTTCATGT-3′
**U6**	Reverse transcribed Primer: 5′-AACGCTTCACGAATTTGCGT-3′
	Forward:5′-CTCGCTTCGGCAGCACA-3′ Reverse:5′-AACGCTTCACGAATTTGCGT-3′

**Table 2:** Primer sequences for quantitative reverse transcription (RT)-PCR (mRNA)

Gene	Sequence (5′ → 3′)
**Human c-Met**	Forward:5′-GTTTCCCAATTTCTGACC-3′ Reverse:5′-TATATCAAAGGTGTTTAC-3′
**Human Bcl-2**	Forward:5′-CTTTGAGTTCGGTGGGGTCA-3′ Reverse:5′-GGGCCGTACAGTTCCACAAA-3′
**Human CyclinD1**	Forward:5′-CTCCTCTCCGGAGCATTTTGATA-3′ Reverse:5′-TTAAAGACAGTTTTTGGGTAATCT-3′
**Human MMP-7**	Forward:5′-GAGTGCCAGATGTTGCAGAA-3′ Reverse:5′-AAATGCAGGGGGATCTCTTT-3′
**Human MMP-9**	Forward:5′-CTGCAGTGCCCTGAGGACTA-3′ Reverse:5′-ACTCCTCCCTTTCCTCCAGA-3′
**Human p57**	Forward:5′-CCCTTCTTCTCGCTGTCCTC-3′ Reverse:5′-CTGGTCCTCGGCGTTCA-3′
**Human GAPDH**	Forward:5′-AGCCTTCTCCATGGTGGTGAA-3′ Reverse:5′-ATCACCATCTTCCAGGAGCGA-3′

### Colony formation assay

Cells were transfected with miR-139-5p mimic or miR mimic NC, miR-139-5p inhibitor or miR inhibitor NC, as described above. Twenty-four hours later, transfected cells were trypsinized, counted and replated at a density of 500 cells/6 cm dish. Ten days later, colonies resulting from the surviving cells were fixed with 3.7% methanol, stained with 0.1% crystal violet and counted. Colonies containing at least 50 cells were scored. Each assay was performed in triplicates.

### Luciferase reporter assays

The 3′-untranslated region (UTR) of human MET was amplified from human genomic DNA and individually inserted into the pmiR-RB-REPORT ™ (Ribobio, Guangzhou, China) using the XhoI and NotI sites. Similarly, the fragment of MET 3′-UTR mutant was inserted into the pmiR-RB-REPORT™ control vector at the same sites. For reporter assays, A549 cells were co-transfected with wild-type (mutant) reporter plasmid and miR-Ribo™ mimics (miR-Ribo™ negative control) using Lipofectamine 2000 (Invitrogen). Firefly and Renilla luciferase activities were measured in cell lysates using the Dual-Luciferase Reporter Assay system. Luciferase activity was measured forty-eight hours post-transfection using dual-glo luciferase reporter system according to the manufacturer's instructions (Promega, Madison, WI, USA). Firefly luciferase units were normalized against Renilla luciferase units to control for transfection efficiency.

The article "Hsa-miR-139-5p inhibits proliferation and causes apoptosis associated with down-regulation of c-Met" was retracted in 2023. Reasons: duplicated images; signs of a paper mill; original data or images not available.

### Transwell migration/invasion assay

A549 and SK-MES-1 cells were grown in RPMI 1640 or DMED containing 10% fetal bovine serum to ~60% confluence and transfected with 50 nM miR-139-5p mimic or a negative control, 100 nM miR-139-5p inhibitor or a negative control. After twenty-four hours, the cells were harvested by trypsinization and washed once with Hanks’ balanced salt solution (Invitrogen). To measure cell migration, 8-mm pore size culture inserts (Transwell; Costar, High Wycombe, UK) were placed into the wells of 24-well culture plates, separating the upper and the lower chambers. In the lower chamber, 500 μL of RPMI 1640 containing 10% FBS was added. Then, serum-free medium containing 5 × 10 4 cells were added to the upper chamber for migration assays, whereas 1 × 105 cells were used for matrigel invasion assays. After twenty-four hours of incubation at 37°C with 5% CO2, the number of cells that had migrated through the pores was quantified by counting 10 independent visual fields under the microscope (Olympus) using *a* × 20 magnifications, and cell morphology was observed by staining with 0.1% crystal violet. Filters were washed thoroughly with 1 × PBS and dissolved in 500 μL of 33% acetic acid, and absorbance was measured at 570 nm. Absorbance of cells incubated in the serum-free medium in the bottom chamber was used as negative control. Each experiment was performed at least three times.

### BrdU immunofluorescence assay

A549 and SK-MES-1 cells were seeded on sterile cover glasses placed in the 6-well plates. After transfection with miR-139-5p mimic, miR mimic NC, miR-139-5p inhibitor, miR inhibitor NC for forty eight hours, the BrdU (5-bromo-2-deoxyuridine; Sigma) stock solution at 10 mg/mL in saline was diluted 1000× in the culture medium and incubated for 60 min. After washing with 1 × PBS, cells were then fixed for 20 min in 4% paraformaldehyde (PFA) and permeabilized with 0.3% Triton X-100 for 10 min. After blocking with 10% goat serum in 1 × PBS for 1 h, cells were incubated with a primary rabbit antibody against BrdU (1:200, Abcam) over night at 4°C, and then incubated with the secondary antibody coupled to a fluorescent marker, Cy3, at room temperature for 2 h. After DAPI staining and 1 × PBS washing, the cover slips were mounted on to glass slides with anti-fade solution and visualized using a fluorescence microscope (Olympus 600 auto-biochemical analyzer, Tokyo, Japan) with Image-Pro Plus software for image analysis, and 10 microscopic fields were taken for calculating BrdU.

The article "Hsa-miR-139-5p inhibits proliferation and causes apoptosis associated with down-regulation of c-Met" was retracted in 2023. Reasons: duplicated images; signs of a paper mill; original data or images not available.

### CCK8 assay

Cell growth was measured using the cell proliferation reagent WST-8 (Roche Biochemicals, Mannheim, Germany). After plating cells in 96-well microtiter plates (Corning Costar, Corning, NY) at 1.0 × 103/well, 10 μL of CCK8 was added to each well at the time of harvest, according to the manufacturer's instructions. One hour after adding CCK8, cellular viability was determined by measuring the absorbance of the converted dye at 450 nm.

### c-Met immunofluorescence assay

A549 cells were seeded on sterile cover glasses placed in the 6-well plates, and then transfected with miR-139-5p mimic, miR mimic NC, miR-139-5p inhibitor, miR inhibitor NC for forty eight hours. After washing with 1× PBS, cells were then fixed for 20 min in 4% paraformaldehyde (PFA) and permeabilized with 0.3% Triton X-100 for 10 min. After blocking with 10% goat serum in 1 × PBS for 1 h, cells were incubated with a primary rabbit antibody against c-Met (1:200, Affinity) over night at 4°C, and then incubated with the secondary antibody coupled to a fluorescent marker, Cy3, at room temperature for 2 h. After DAPI staining and 1 × PBS washing, the cover slips were mounted on to glass slides with anti-fade solution and visualized using a fluorescence microscope (Olympus 600 auto-biochemical analyzer, Tokyo, Japan) with Image-Pro Plus software for image analysis.

### Transfection of siRNA

Three siRNA duplexes targeting human MET mRNA (GenBank accession no. NM_014033) were designed and synthesized by Guangzhou RiboBio Company (Guangzhou, China). For transfection, the cells were plated on an antibiotic-free growth medium at 30–40% confluence approximately 24 h before transfection. RNA oligonucleotides were transfected at a final concentration of 50 nM, using Lipofectamine 2000 (Invitrogen, USA) according to the manufacturer's protocol.

### Tumor formation in BALB/c nude mice

BALB/c athymic nude mice (male, 4–6-weeks old and 16–20 g) were purchased from Hubei Research Center of Laboratory Animal (Wuhan, China). All animal experiments were carried out in accordance with the Guide for the Care and Use of Laboratory Animals of Wuhan University. To establish lung cancer xenograft model, 5 × 105 A549 cells were suspended in 100 μL phosphate-buffered saline and inoculated subcutaneously into the flanks of nude mice. After 8 days, the transplanted nude mice were randomly divided into two groups (*n* = 6 each). MiR-139-5p agomir (miR-139-5p) or miR agomir NC (NC) (RiboBio Co., Ltd, Guangzhou, China) was directly injected into the implanted tumor at the dose of 1 nmol (in 20 μL phosphate-buffered saline) per mouse every 4 days for seven times. The tumor size was monitored by measuring the length (L) and width (W) with calipers every 4 day, and the volumes were calculated using the formula: (L × W2)/2. Mice were killed by cervical dislocation in day 28, and the tumors were excised and snap-frozen for protein and RNA extraction.

The article "Hsa-miR-139-5p inhibits proliferation and causes apoptosis associated with down-regulation of c-Met" was retracted in 2023. Reasons: duplicated images; signs of a paper mill; original data or images not available.

### Hoechst 33342 staining

Apoptotic morphological changes in the nuclear chromatin of cells were detected by Hoechst 33342 staining. A549 and SK-MES-1 cells were seeded on sterile cover glasses placed in the 6-well plates. After overnight growth, cells were transfected with miR-139-5p mimic, miR mimic NC, miR-139-5p inhibitor and miR inhibitor NC for forty eight hours. Then cells were washed with phosphate-buffered saline (PBS) and fixed with 4% PFA for 10 min, and then incubated with 5 ug/mL Hoechst 33342 staining solution for 10 min. After three washes with 1× PBS, the cells were viewed and recorded by Image-Pro Plus software (Media Cybernetics, Silver Spring, MD) under a fluorescence microscope (Olympus 600 auto-biochemical analyzer, Tokyo, Japan).

### Annexin V-FITC/PI analysis

A549 cells were seeded on sterile cover glasses placed in the 6-well plates. After overnight growth, cells were transfected with miR-139-5p mimic, miR mimic NC, miR-139-5p inhibitor and miR inhibitor NC for forty eight hours. Then cells were washed with 1 × PBS and fixed with 4% PFA for 10 min, and then incubated with Annexin V-FITC and Propidium (BestBio, Shanghai, China) following the manufacturer's instructions. Then they were finally observed under fluorescence microscopy (Olympus 600 auto-biochemical analyzer, Tokyo, Japan). Using Image-Pro Plus software (Media Cybernetics, Silver Spring, MD) to record images and analyze cell apoptosis.

### Flow cytometry

A549 cells transfected with miR-139-5p mimic or negative control were trypsinized and resuspended in 1 × binding buffer at 1 × 106 cells/mL. 100 μL of this cell suspension was incubated with 5 μL of FITC-Annexin V and 5 μL propidium iodide (PI) for 15 minutes in the dark. The reaction was terminated with the addition of 400 μL 1 × binding buffer and analyzed with (FACSCalibur using the CellQuest software (Becton Dickinson). FITC-Annexin V-positive and PI-negative cells were considered as apoptotic and the experiments were carried out in triplicates.

### Wound healing assay *in vitro*

The A549 cells were seeded in 6-well plates and incubated for twenty-four hours. Then a linear wound was created by dragging a 1-mL pipette tip through the monolayer prior to transfection. Cellular debris was removed by gentle washes with culture medium, following which transfection was performed immediately, and the cells were allowed to migrate for a further forty-eight hours. The healing process was dynamically photographed after the wound was introduced using a microscope (Olympus 600 auto-biochemical analyzer, Tokyo, Japan). Migration distance was measured from images (5 fields) taken at each indicated time point. The gap size was analyzed using Image-Pro Plus 6.0 software. The residual gap between the migrating cells from the opposing wound edge was expressed as a percentage of the initial gap size.

The article "Hsa-miR-139-5p inhibits proliferation and causes apoptosis associated with down-regulation of c-Met" was retracted in 2023. Reasons: duplicated images; signs of a paper mill; original data or images not available.

### Caspase-3 activity assay

The activity of caspase-3 was determined using the caspase-3 activity kit (Beyotime Institute of Biotechnology, Haimen, China). To evaluate the activity of caspase-3, cell lysates were prepared after their respective treatment with various designated treatments. Assays were performed on 96-well microtitre plates by incubating 10 μL protein of cell lysate per sample in 80 μL reaction buffer (1% NP-40, 20 mM Tris-HCl (pH 7.5), 137 mM Nad and 10% glycerol) containing 10 μL caspase-3 substrate (Ac-DEVD-pNA) (2 mM). Lysates were incubated at 37°C for 4 h. Samples were measured with an ELISA reader at an absorbance of 405 nm. The detail analysis procedure was described in the manufacturer's protocol.

### Statistical analysis

All experiments were repeated 3 times independently. The results are presented as the means ± standard error mean (SEM). A two-tailed paired *t*-test and One-way ANOVA were performed using SPSS 19.0 software in order to detect significant differences in measured variables between groups. A value of *P* < 0.05 was considered to indicate a statistically significant difference.

## SUPPLEMENTARY MATERIALS FIGURES



## Abbreviations

miR: microRNA
miR-139-5p: hsa-microRNA-139-5p
NSCLC: non-small cell lung cancer
3′-UTR: 3′-untranslated region
ER: estrogen receptor alpha
BCL2: B-cell lymphoma-2
